# Enhanced Inhibitory Effect of DC-CIK Cells on Lung Adenocarcinoma via Anti-Tim-3 Antibody and Antiprogrammed Cell Death-1 Antibody and Possible Mechanism

**DOI:** 10.1155/2022/4097576

**Published:** 2022-07-31

**Authors:** Liang Zhou, Qijiu Chen, Hui Chen, Li Wang, Jianyong Zhang

**Affiliations:** ^1^The Second Department of Respiratory and Critical Care Medicine, Affiliated Hospital of Zunyi Medical University, Zunyi 563000, Guizhou, China; ^2^Department of Respiratory and Critical Care Medicine, The Fifth Affiliated Hospital of Sun Yat-sen University, Zhuhai 519000, Guangdong, China; ^3^Key Laboratory of Cell Engineering in Guizhou Province, Affiliated Hospital of Zunyi Medical University, Zunyi 563000, Guizhou, China

## Abstract

**Objective:**

To investigate the effect and mechanism of blocking the signaling pathways of the T-cell immunoglobulin and mucin domain-containing protein 3 (Tim-3) and programmed death protein 1 (PD-1) in dendritic cell-cytokine induced killer (DC-CIK) cells on human lung adenocarcinoma A549 cells.

**Methods:**

Peripheral blood mononuclear cells (PBMCs) were isolated and induced into mature DC-CIK cells by cytokines *in vitro*. After blocking the Tim-3 and PD-1 signaling transduction pathways with anti-Tim-3 and anti-PD-1 antibodies, DC-CIK cells were coincubated with A549 cells. The killing effect of DC-CIK cells against A549 cells was measured by a CCK-8 assay. The impact of DC-CIK cells on the invasion and migration ability of A549 cells was detected by the Transwell test. The apoptosis rate of DC-CIK cells and the ratio of CD4^+^, CD8^+^, and DC-CIK cell subsets were determined by flow cytometry. The cell proliferation of DC-CIK was detected by the CCK-8 assay.

**Results:**

The antibodies of anti-Tim-3 antibody and anti-PD-1 could block Tim-3^+^ and PD-1^+^ DC-CIK cells and could significantly increase the killing effect of DC-CIK cells on A549 cells. The number of A549 cells under the microporous membrane of the Transwell chamber was reduced considerably in invasion and migration tests. Anti-Tim-3 and anti-PD-1 antibodies significantly reduced apoptosis of DC-CIK cells. No significant differences were observed in the ratios of CD4^+^ and CD8^+^ DC-CIK cell subsets or the proliferation capacity of DC-CIK cells in each group.

**Conclusion:**

Blocking the Tim-3 and PD-1 signaling pathways of DC-CIK cells with antibodies can enhance the killing ability of DC-CIK cells in A549 cells and significantly suppress the invasion and migration ability of A549 cells. The potential mechanism may be related to reduced apoptosis of DC-CIK cells.

## 1. Introduction

Lung cancer is a type of malignant tumor that has the highest rates of morbidity and mortality worldwide. Lung cancer is common and the primary cause of cancer death in China, with 733,000 newly diagnosed cases a year, and the 5-year survival rate is 16.1% [1–3]. Lung cancer has been considered one of the life-threatening malignant tumors. With the development of molecular biology and tumor immunology, tumor immunotherapy has revealed an encouraging effect in treating various malignant tumors following traditional surgical treatment, radiotherapy, or chemotherapy. Immunotherapy significantly prolongs survival and improves the quality of life in patients with lung cancer. Immunotherapy aims to adjust the balance between body immunity and tumors by regulating the body's immune response, directly killing tumor cells, and interfering with tumor biological behaviors, such as tumor growth, differentiation, apoptosis, invasion, and metastasis. Immunotherapy modalities contain mainly immune checkpoint inhibitors (ICIs), adoptive cellular immunotherapy (ACI), and tumor vaccines. The programmed death protein 1 (PD-1) inhibitors are one of the representatives of ICIs. Dendritic cell-cytokine-induced killer cells (DC-CIK) are *in vitro* induced immune effector cells with specific tumoricidal activity. The pronounced antitumor effect of DC-CIK cells in multiple tumors has been reported [4]. The possible reasons may be associated with the cell surface expressions of the T cell immunoglobulin, the programmed death protein 1 (PD-1), mucin domain-containing protein 3 (Tim-3), and other negative-regulatory factors [5–8].

Tim-3 is a crucial negative costimulatory molecule that has emerged recently, except that blocking PD-1/PD-L1 can produce a good antitumor effect. Tim-3 belongs to the T-cell immunoglobulin and mucin domain protein family that contains eight members (Tim-1 to Tim-8). However, only Tim-1, Tim-3, and Tim-4 exist in humans. Tim-3 is a single-transmembrane protein with an IgV subunit, a mucin-like domain, a single-transmembrane domain, and a Tyr-rich intracellular domain from the N- to C-terminus of the peptide chain. Galectin-9 (Gal-9) is a ligand for Tim-3, and its binding to Tim-3 can stimulate intracellular signaling pathways [9]. Tim-3 is expressed on the surface of Th1 cells, Tcl cells [10], Th17 cells, NK cells, monocytes, macrophages, DC cells, and other immune cells [11, 12]. It is believed that Tim-3 has an essential impact on immune responses in intracellular infection, tumor immunity, and autoimmune diseases [13]. Tim-3 can induce a tumor microenvironment dominated by immunosuppression by functional suppression and exhaustion of T cells and synergistic expressions of Foxp3, CTLA-4, and other harmful immunoregulatory molecules to further attenuate the function of T cells in tumor-killing [14]. The anti-Tim-3 antibody can promote the IFN release of IFN-*γ* in T cells. It can therefore regulate antitumor immunity and suppress breast cancer, colorectal cancer, prostate cancer, etc. [15]. In addition, Tim-3 and PD-1 are often co-expressed on the T-cell surface. Double-positive Tim-3 and PD-1 T cells are associated with more severe exhaustion and weaker cytokine secretory capacity than PD-1 single-positive T cells [16].

Our study investigated whether anti-Tim-3 and anti-PD-1 antibodies could enhance the tumor-specific immune response of DC-CIK cells and produce a more substantial tumor-killing effect by blocking the cell surface Tim-3 and PD-1 signaling pathways. The findings could provide new strategies for optimizing immunotherapy for lung cancer.

## 2. Materials and Methods

### 2.1. Materials and Reagents

Fresh peripheral blood samples were collected from healthy volunteers. The human lung cancer cell line A549 was derived from the passaged cell line preserved in the immunology laboratory of Zunyi Medical University. Tim-3 blocking antibody (AB_1877089) and PD-1 blocking antibody (AB_2820104) were purchased from Biolegend Inc., USA. The cell factors rhIL-4, rhGM-CSF, rhIFN-*γ*, rhTNF-*α*, and CD3McAb were purchased from Peprotech Inc., USA. Flow cytometry antibodies CD3-PE-Cy5, CD56-RD1, CD4-FITC, CD8-PC-Cy7, Tim-3-APC, and PD-1-PE were purchased from BD Inc., USA. The 1640 medium was purchased from Thermo Scientific Inc., USA. The GTT-551 H3 medium was from TaKaRa Company, Dalian, China.

### 2.2. Cultivation of Mature DC Cells

Peripheral blood mononuclear DC cells were isolated from healthy volunteers by density gradient centrifugation. Isolated cells were incubated in a 1640 medium for two hours at 37°C. The incubation was then continued in a GTT-551 H3 medium that contained 5% autologous serum, rhIL-4 (500 U/mL), and rhGM-CSF (1000 U/mL). The fluid medium was renewed and re-added with cytokines on day 3. Antigen A549 (50 *μ*g/mL) was added to stock DC cells on day 5. DC cell maturation was induced by adding rhTNF-*α* (20 ng/mL) on day 6. Mature DC cells were harvested on day 7.

### 2.3. Induction and Cultivation of DC-CIK Cells

DC-CIK peripheral blood mononuclear cells were isolated from healthy volunteers by density gradient centrifugation. The isolated cells were incubated in a serum-free medium supplemented with rhIFN-*γ* (1000 U/ml) on day 0, and with CD3McAb (50 ng/mL) and rhIL-2 (1000 U/mL) after 24 hours. The fluid medium was double replenished or half replenished every three days according to the cell state and the color of the medium, and rhIL-2 (1000 U/mL) was added in either situation. A549 antigen-loaded adherent DC cells were suspended by gently pipetting with a pipette on day 7. The DC cells were co-incubated with CIK cells in a ratio of 1∶10 to harvest mature DC-CIK cells. The proportions of CD3^+^, CD56^+^, CD4^+^, CD8^+^, Tim-3^+^, and PD-1^+^ DC-CIK cells were detected by flow cytometry.

### 2.4. Blockade of Tim-3 and PD-1 with Antibodies and Evaluation of the Blocking Effect

DC-CIK cells were collected with a concentration adjusted to 1 × 10^6^/mL and divided into a blank control group, a Tim-3 blockade group, a PD-1 blockade group, and a Tim-3^+^PD-1 blockade group. Cells were not treated in the blank control group. In contrast, those in the Tim-3 blockade group, the PD-1 blockade group, and the Tim-3^+^PD-1 blockade group were added with anti-Tim-3 blocking antibody (10 *μ*g/mL), anti-PD-1 blocking antibody (10 *μ*g/mL), and anti-Tim-3 antibody (10 *μ*g/mL) plus anti-PD-1 blocking antibody (10 *μ*g/mL), respectively. After incubation at 37°C under 5% CO^2^ for one hour, the cell suspension was washed three times with PBS to remove residual antibodies and resuspended in a complete medium for further experiment. The ratios of Tim-3^+^ and PD-1^+^ DC-CIK cells were again measured.

### 2.5. CCK-8 Assay for Analyzing the Killing Effect of DC-CIK Cells on A549 Cells

DC-CIK cells in each group were incubated with A549 cells in an effector to target ratios of 10 : 1, 20 : 1, and 30 : 1 in a 37°C incubator with 5% CO^2^. Incubation was terminated after six hours. A CCK-8 solution was added at a dose of 10 *μ*L to each well over two hours. The killing activity of CIK cells was detected by measuring the absorbance at 450 nm using a microplate reader [17].

### 2.6. Transwell Test for Analyzing the Effect of DC-CIK Cells on the Invasion and Migration Capacity of A594 Cells

Matrigels were liquefied and diluted in a 1 : 4 ratio before being added to a Transwell chamber. The basement membrane was hydrated at room temperature. After a 12-hour withdrawal of serum starvation, A549 cells were added to a Matrigel-coated Transwell chamber and co-incubated with DC-CIK cells in each group for 24 hours. The chamber was removed, washed with PBS to carefully remove cells in the microporous inner membrane using a cotton swab, fixed in 95% alcohol for five minutes, and dyed with 4 g/L crystal violet. Cells that migrated to the microporous sublayer membrane were counted under a microscope. The average counts in ten fields, which were randomly selected, were imaged and recorded for each sample.

### 2.7. Flow Cytometry to Measure Apoptosis of DC-CIK Cells

DC-CIK cells were resuspended in each group in 1 × binding buffer and incubated in the dark with AnnexinV-FITC for 10 minutes and propidium iodide for five minutes. Cells were tested on the flow cytometer after vigorous mixing in a 1 × binding buffer.

### 2.8. Flow Cytometry to Measure the Ratio of CD4^+^ and CD8^+^ DC-CIK Cells

DC-CIK cells in each group were resuspended in PBS and incubated with the CD4-FITC and CD8-PC-Cy7 antibodies at room temperature in the dark for 25 minutes. After rinsing with the flow cytometry washing solution, the cells were resuspended in PBS and were detected on the flow cytometer.

### 2.9. CCK-8  Assay for Determining Proliferation Activity of  DC-CIK Cells

DC-CIK cells in each group were seeded on the 96-well plate and placed in a 37°C, 5% CO^2^ incubator. CCK-8 reagent was added at 0, 24, 48, and 72 hours, to incubate for two hours. The optical density (OD) at 450 nm was determined by the enzyme-linked immunosorbent assay. The cell growth curve over time was drawn.

### 2.10. Statistical Methods

All statistical analyses were conducted using GraphPad Prism 8 and SPSS 22.0 software. Continuous variables were expressed as $\bar{x}\pm s$. Two sets of data were compared by *t*-test. A one-way analysis of variance (ANOVA) with an LSD posthoc test was applied to compare multiple data sets. A *P* value below 0.05 was considered to be statistically significant.

## 3. Results

### 3.1. Morphology of DC-CIK Cells

A549 cells grew naturally with a triangular, short fusiform or polygonal shape, a distinct border, a plump appearance, a smooth surface, a consistent refractive index, a large nucleus, and a prominent nuclear membrane and nucleolus outline. The extension of pseudopodia-like protrusion at the cell periphery and the intercellular junction was identified in low-density areas (Figure 1(a)).

DC cells demonstrated adherent growth with a round shape and smooth contour on day 0. Cells started to enlarge with an irregular round shape, and burr-like protrusions appeared at the cell periphery within 2-3 days. There were apparent synapse-like structures in the cell periphery at 4–6 days. Some cells showed simultaneous suspension growth, among which a small proportion aggregated into clusters (Figure 1(b)). After the addition of TNF-*α*, most cells showed suspension growth with typical burr-shaped protrusions in the periphery of the cell for 7-8 days (Figure 1(b)).

After incubation on day 0, the CIK cells were round and translucent in an evenly suspended state. On day 3, small clusters of cells grown in grape-shaped clusters were found. The clustered cells were round and regular at high density, whereas the dispersed cells were round and translucent with a consistent refractive index. The co-incubated CIK and DC cells demonstrated no changes in morphology and started to increase massively at 7–12 days. Cell growth remained in clusters. Dispersed cell clusters were also observed. After the dispersal process, the cells were found to be round and plump with high transmittance, and tiny rough tentacles appeared on the cell surface. CIK cell proliferation was slow at 1–7 days, became faster after that, and expanded approximately 100 times on day 14 (Figure 1(c)).

### 3.2. Phenotypes of DC-CIK Cells

DC-CIK cells derived from PBMCs were induced and amplified. In analyses of DC-CIK cell phenotypes by flow cytometry, the ratios of CD3^+^T cells, CD3^+^CD56^+^NKT cells, CD3-CD56^+^NK cells, CD4^+^helper/inducer T cells, and CD8^+^cytotoxic/suppressor T cells were 10.55% ± 5.90, 4.00% ± 1.62, 22.76% ± 1.90, and 74.22% ± 4.78, respectively (Figure 2).

### 3.3. Blocking Effect of Anti-Tim-3 and Anti-PD-1 Antibodies in DC-CIK Cells

The ratios of Tim-3^+^ DC-CIK cells, PD-1^+^ DC-CIK cells, and Tim-3^+^PD-1^+^ DC-CIK cells were 78.76% ± 10.20, 5.76% ± 6.90, and 11.22% ± 7.42, respectively, before adding antibodies. The ratios of Tim-3^+^ DC-CIK cells and PD-1^+^ DC-CIK cells decreased to 0.39% ± 0.17 and 0.11% ± 0.09, respectively, after the use of TIM-3 and PD-1 blocking antibodies, suggesting an excellent blocking effect of the antibody specific for Tim-3 and PD-1 (Figure 3).

### 3.4. Killing Effect of  DC-CIK Cells on A549 Cells in Each Group

In the analysis of morphological changes, DC-CIK cells co-incubated with A549 cells were observed under an inverted microscope. As a result, directional aggregations of CIK cells were observed around A549 cells and were in a typical rosette form. Fine particles appeared in the cytoplasm of A549 cells that gradually blurred and disappeared, leaving massive cell fragments in the middle of the medium. In contrast, A549 cells in the control group had adherent growth and continued to increase. Separately incubated DC-CIK cells were evenly distributed throughout the field of view and clustered or clumped in grape-like shapes. An analysis of tumor-killing activity revealed that the killing activity of DC-CIK cells in the four groups improved significantly as the ratio of effectors to target cells increased. At an effector-to-target ratio of 20 ∶ 1, the killing activity of DC-CIK cells in the Tim-3 blockade group, PD-1 blockade group, and Tim-3^+^PD-1 blockade groups was significantly higher than that in the blank control group (*P* < 0.05) (Figure 4). At an effector-to-target ratio of 30 ∶ 1, the killing activity of DC-CIK cells in the Tim-3 blockade group and the PD-1 blockade group was remarkably higher than that in the blank control group (*P* < 0.05) (Figure 4). There were no significant differences in the killing activity of DC-CIK cells on A549 cells between the Tim-3 blockade group, the PD-1 blockade group, and the Tim-3^+^PD-1 blockade group (Table 1).

### 3.5. Effect of DC-CIK Cells on the Invasion and Migration Capacity of  A549 Cells in Each Group

The Transwell invasion assay was performed to compare the invasion (Figure 5, Table 2) and migration (Figure 6, Table 3) ability of A549 lung adenocarcinoma cells in the blank control group, the Tim-3 blockade group, the PD-1 blockade group, and the Tim-3^+^PD-1 blockade group. After coincubation for 24 hours, the number of A549 cells in the Tim-3 blockade group, the PD-1 blockade group, and the Tim-3^+^PD-1 blockade group was significantly reduced compared to the blank control group (*P* < 0.05). Simultaneously, the A549 cells in the Tim-3 blockade group and the PD-1 blockade group were also less than those of the Tim-3+PD-1 blockade group (*P* < 0.05). Consequently, a single or combined blockade of Tim-3 and PD-1 could significantly enhance the inhibitory effect of DC-CIK cells on the invasion ability of lung adenocarcinoma A549 cells. Still, the simultaneous blockade of Tim-3 and PD-1 did not produce an apparent synergistic effect.

### 3.6. Detection of Apoptosis of DC-CIK Cells in Each Group

After blocking with the antibody for 24 hours, DC-CIK cells in each group were analyzed for apoptosis by flow cytometry using Annexin V-FITC and PI staining. The flow cytometry chart (Figure 7) shows necrotic cells in the upper left quadrant (Annexin V^−^/PI^+^), normal cells in the lower left quadrant (Annexin V^−^/PI^−^), late apoptotic cells in the upper right quadrant (Annexin V^+^/PI^+^), and early apoptotic cells in the lower right quadrant (Annexin V^+^/PI^−^). Further analysis of the data is shown in Figure 7, Table 4. The apoptosis rate of DC-CIK cells in the Tim-3 blockade group and the Tim-3^+^PD-1 blockade group was significantly reduced compared with that in the blank control group (*P* < 0.001). At the same time, the apoptotic rate in the Tim-3^+^PD-1 blockade group was notably less than that of the Tim-3 blockade group (*P* < 0.05). A significantly reduced apoptotic rate was also observed in the Tim-3 blockade group and the Tim-3^+^PD-1 block group compared to the PD-1 blockade group (*P* < 0.01).

### 3.7. Ratio of CD4^+^ and CD8^+^ DC-CIK Cells in Each Group

Given the pivotal role of CD4^+^ and CD8^+^ DC-CIK cells in tumor immunity, the effect of the Tim-3 and PD-1 blockades on the function of DC-CIK cells was explored by determining the expression rate of CD4^+^ and CD8^+^ DC-CIK cells in the Tim-3 blockade group, the PD-1 blockade group, and the Tim-3^+^PD-1 blockade group. The results showed that the ratios of the CD4^+^ and CD8^+^ DC-CIK cell subsets were not significantly different between the Tim-3 blockade group, the PD-1 blockade group, and the Tim-3^+^PD-1 blockade group (*P* > 0.05). The findings suggested that blocking the expression of Tim-3 and PD-1 on the surface of DC-CIK cells did not affect the ratio of DC-CIK cell subsets (Figures 8(a)and 8(b), Table 5).

### 3.8. Detection of DC-CIK Cell Growth in Each Group

The CCK-8 assay measured the OD value of DC-CIK cells in each group at 0–3 days. DC-CIK cells in each group were calculated on the standard curve to draw a growth curve. The number of DC-CIK cells increased with time and showed no significant differences within groups. Such results suggested that the addition of the anti-Tim-3 antibody and anti-PD-1 antibody had no apparent effect on DC-CIK cell growth (Figure 8(c)).

## 4. Discussion

Due to the annual increase in incidence and high mortality, lung cancer has become one of the most common malignant tumors that threaten human health in the world. Immunotherapy regulates the body's immune response and has revealed an encouraging effect in treating lung cancer. ICIs is one type of immunotherapy. As a representative drug of ICIs, nivolumab enhances the function of T cells that are essential in tumor immunity by blocking the PD-1/programmed death-ligand 1 (PD-L1) pathways [18]. The process mobilizes the body's immune system against tumors to significantly prolong the overall survival (OS) of patients with lung cancer [18–21]. However, the existing monotherapies have problems such as easy tumor recurrence. Exploring a safe therapy that can produce a long-lasting antitumor effect, avoid the risk of recurrence, and provide good compliance and safety is a consistent goal in treating advanced non-small-cell lung cancer (NSCLC). The regimen that combines ICI therapy with chemotherapy or targeted therapy is proposed by researchers and exhibits some advantages in triple-negative breast cancer, lung cancer, and renal cell carcinoma. However, the desired therapeutic effect is not achieved considering the severity of adverse reactions in some patients [22–26]. Another regimen is the combined use of two types of ICI, which has achieved promising results in some patients with NSCLC, melanoma, and renal cell carcinoma [27, 28].

Tim-3 is a crucial negative costimulatory molecule that has emerged recently. The anti-Tim-3 antibody can promote the IFN release of IFN-*γ* in T cells. It can therefore regulate antitumor immunity. In addition, Tim-3 and PD-1 are often co-expressed on the T-cell surface. Double-positive Tim-3 and PD-1 T cells are associated with more severe exhaustion and weaker cytokine secretory capacity than PD-1 single-positive T cells [16]. In a mouse model of lung adenocarcinoma, Tim-3 was found to be a targetable biomarker that may be related with adaptive resistance to inhibition of PD-1 [29]. Double blocking of Tim-3 and PD-1 can improve the tumor immunosuppression microenvironment. Tim-3 appears to be a promising target for ICI therapy, and its combination with PD-1 blockers may show a better antitumor effect.

ICI therapy depends on the patient's own preexisting endogenous antitumor immunity. However, many cancer patients cannot generate a reliable antitumor immune response, especially those receiving high-dose chemotherapy, which even leads to the collapse of the immune system [30, 31]. ICI achieves the antitumor effect by infusing immune cells with antitumor activity into tumor patients to directly kill or activate the body's immune response [32]. Thus, combining ICI and activated immune effector cells has been hypothesized to produce a potent antitumor effect for cancer patients, including those with immune dysfunction. DC-CIK cells are immune effector cells mediated *in vitro* with specific antitumor activity, which achieve the antitumor result by releasing NKG2D-mediated perforin and eliciting Fas/FasL-mediated apoptosis of tumor cells [33]. Clinical studies have confirmed a strong antitumor activity of DC-CIK cells in various tumors [4]. For PD-1 and Tim-3, which are also expressed on the surface of DC-CIK cells, their ability to kill tumors can be significantly enhanced by blocking the PD-1 signaling pathway [5–7]. A clinical remission rate of 64.5% with no apparent side effects is reported when DC-CIK cells incubated with an anti-PD-1 antibody are used to treat solid advanced tumors such as lung and liver tumors [31]. Therefore, combining ICI with DC-CIK cells during incubation or after infusion may have potent antitumor effects in treating tumor patients, which includes the immunocompromised.

Our study extracted peripheral blood PBMCs and induced them into DC-CIK cells. Tim-3 and PD-1 expressed on the surface of DC-CIK cells were blocked with a specific antibody to block the adverse regulatory pathways between DC-CIK cells and tumor cells. Our study revealed that a blockade of Tim-3 and PD-1 expressions on the surface of DC-CIK cells could significantly enhance their direct killing effect on lung adenocarcinoma, suppressing the invasion and migration ability of lung adenocarcinoma substantially and enhancing their antitumor activity. To further analyze the mechanism of action, we found that the apoptotic rate of DC-CIK cells fell after the Tim-3 blockade but did not change significantly after the single blockade of PD-1. Furthermore, the combined blockade of PD-1 with Tim-3 significantly suppressed DC-CIK cells better than the single blockade of Tim-3. Previous studies have demonstrated that apoptosis of CD8^+^ T cells is accelerated by eliciting the expression of PD-L1 in hepatoma cells in an IFN-*γ*-dependent way [34].

In contrast, early apoptosis of CD8^+^ T cells is suppressed by blocking the Tim-3 pathway [35]. Functional improvement in DC-CIK cells through blockade of Tim-3 and PD-1 signal transduction pathways may be involved in the apoptotic pathways. In our study, the cell proliferation test showed that blocking Tim-3 and PD-1 on the surface of DC-CIK cells had no significant effect on their proliferation. The findings may be related to the specificity of the DC-CIK cell population or the lack of substantial differences in the small sample size. Hence, much deeper research is required.

Blocking Tim-3 and PD-1 extends the action time of DC-CIK cells *in vivo* to achieve a long-lasting antitumor effect. Meanwhile, combining Tim-3 and PD-1 blocking antibodies with DC-CIK cells *in vitro* before administration to tumor patients can mitigate the impact of ICI on normal cells and the body's immune system and further reduce immune-related side effects during treatment. A series of studies have confirmed that DC-CIK cell infusion is responsible for mild and transient fever without any other apparent toxic response and improves chemotherapy/radiation therapy-related leukopenia, gastrointestinal adverse reactions, anemia, and liver dysfunction [36, 37].

In summary, our study confirms that blocking the Tim-3 signaling transduction pathway in DC-CIK cells with an anti-Tim-3 antibody can improve the tumoricidal effect of DC-CIK cells through *in vitro* experiments. Still, *in vivo* experimental studies are required for further verification. With the in-depth research into tumor molecular biology, combination therapy using ICI and DC-CIK cells is expected to become a potential optimization immunotherapy.

## Figures and Tables

**Figure 1:** (a) Morphology of A549 cells. (b) Morphology of DC cells. (c) Morphology of DC-CIK cells.

**Figure 2:** Cell phenotype of DC-CIK. (a) Flow sorting chart. (b) Statistics chart.

**Figure 3:** (a) Cell ratio of Tim-3^+^ DC-CIK before blocking DC-CIK with anti-Tim-3 antibody. (b) Cell ratio of PD-1^+^ DC-CIK before blocking DC-CIK with anti-PD-1 antibody. (c) Cell ratio of Tim-3^+^ PD-1^+^ DC-CIK before blocking DC-CIK with anti-Tim-3 antibody and anti-PD-1 antibody. (d) Cell ratio of Tim-3^+^ DC-CIK after blocking DC-CIK with anti-Tim-3 antibody. (e) Cell ratio of PD-1^+^ DC-CIK after blocking DC-CIK with anti-PD-1 antibody. (f) The proportion of different cell phenotypes ^*∗∗*^*P* < 0.001.

**Figure 4:** Killing rate of DC-CIK cells in different groups against A549 cells ^*∗*^*P* < 0.05.

**Figure 5:** Invasion of cells in the microporous membrane of the Transwell chamber. (a) Cell morphology across the chamber. (b) Statistics chart ^*∗*^*P* < 0.05.

**Figure 6:** Migration of cells in the microporous membrane of the Transwell chamber. (a) Cell morphology across the chamber. (b) Statistics chart ^*∗*^*P* < 0.05.

**Figure 7:** (a) Apoptotic rate of DC-CIK cells in the blank control group. (b) Apoptotic rate of DC-CIK cells in the Tim-3 blockade group. (c) Apoptotic rate of DC-CIK cells in the PD-1 blockade group. (d) Apoptotic rate of DC-CIK cells in the Tim-3 +PD-1 blockade group. (e) Statistics chart ^*∗*^*P* < 0.01; ^&^*P* < 0.05.

**Figure 8:** (a) Proportion of CD4^+^ DC-CIK cells. (b) Proportion of CD8^+^ DC-CIK cells. (c) Cell viability curve of DC-CIK in different groups. ^NS^*P* < 0.05.

**Table 1:** The killing rate of DC-CIK cells in different groups against A549 cells under different target ratios ($\bar{x}\pm s$,%).

Target effect ratio	Control	Tim-3 block	PD-1 block	Tim-3+PD-1 block
10 : 1	29.38 ± 9.89	27.89 ± 5.38	31.43 ± 7.67	33.45 ± 8.52
20 : 1	38.06 ± 3.64	59.89 ± 8.71^*∗*^	57.64 ± 7.62^*∗*^	57.93 ± 8.27^*∗*^
30 : 1	51.49 ± 7.30	74.19 ± 11.03^*∗*^	71.86 ± 14.89^*∗*^	67.28 ± 7.58

*Note.* Compared with the blank control group, ^*∗*^*P* < 0.05.

**Table 2:** The invasion of cells in the microporous membrane of the Transwell chamber ($\bar{x}\pm s$).

Group	Number of Cells (per/high magnification)
Blank control	82.60 ± 9.31
Tim-3 block	19.20 ± 8.89^*∗*^^#^
PD-1 block	19.40 ± 7.86^*∗*^^#^
Tim-3+PD-1 block	32.60 ± 6.36^*∗*^

*Note.* Compared with the blank control group, ^*∗*^*P* < 0.0001; compared with the Tim-3+PD-1 blocking group, ^#^*P* < 0.05.

**Table 3:** The cells in the Transwell chamber microporous membrane ($\bar{x}\pm s$).

Group	Number of cells (per/high magnification)
Blank control	105.00 ± 6.00
Tim-3 blockade	63.00 ± 8.51^*∗*^
PD-1 blockade	66.40 ± 7.83^*∗*^^#^
Tim-3^+^PD-1 blockade	55.80 ± 6.38^*∗*^

*Note.* Compared with the blank control group, ^*∗*^*P* < 0.0001; compared with the Tim-3+PD-1 blockade group, ^#^*P* < 0.05.

**Table 4:** The apoptotic rate of DC-CIK cells in different groups ($\bar{x}\pm s$).

Group	DC-CIK apoptosis rate of cells (%, $\bar{x}\pm s$)
Blank control	6.54 ± 1.23^&^
Tim-3 blockade	2.91 ± 0.79^*∗*^^#^
PD-1 blockade	8.25 ± 1.17^&^
Tim-3+PD-1 blockade	0.23 ± 0.05^*∗*^^#&^

*Note.* In comparison with the blank control group, ^*∗*^*P* < 0.0001; in comparison with the PD-1 blockade group, ^#^*P* < 0.01; in comparison with the Tim-3 blockade group, and *P* < 0.05.

**Table 5:** The cell phenotype of DC-CIK in different groups after blocking ($\bar{x}\pm s$).

Group	CD4^+^	CD8^+^
Blank control	4.23 ± 0.79	93.54 ± 0.64
Tim-3 blockade	3.86 ± 1.20	93.59 ± 1.75
PD-1 blockade	4.15 ± 1.01	93.59 ± 0.83
Tim-3+PD-1 blockade	3.80 ± 1.15	94.22 ± 1.25

## Data Availability

All data generated or analyzed during this study are included in this published article.
